The article "Identification of Serum Metabolomics Characteristics in Patients with Stable Angina Pectoris Using UHPLC-QE-MS" was retracted in 2023. Reasons: suspected computer-generated content; unreliable results or conclusions; concerns about the data; concerns about the results or conclusions.

# Identification of Serum Metabolomics Characteristics in Patients with Stable Angina Pectoris Using UHPLC-QE-MS

**DOI:** 10.1155/2022/3900828

**Published:** 2022-05-16

**Authors:** Yufei Zhou, Chen Zhou, Gang Luo, Wei Ren, Li Dong, Junjie Liang, Linshen Mao, Mengnan Liu, Yanli Dong, Pan Liang, Sijin Yang

**Affiliations:** ^1^National Traditional Chinese Medicine Clinical Research Base and Cardiovascular Medicine Department of the Affiliated Traditional Chinese Medicine Hospital of Southwest Medical University, Luzhou, 646000 Sichuan, China; ^2^College of Integrated Traditional Chinese and Western Medicine, Southwest Medical University, Luzhou, 646000 Sichuan, China; ^3^National Traditional Chinese Medicine Clinical Research Base and Drug Research Center of the Affiliated Traditional Chinese Medicine Hospital of Southwest Medical University, Luzhou, 646000 Sichuan, China; ^4^Faculty of Chinese Medicine and State Key Laboratory of Quality Research in Chinese Medicine, Macau University of Science and Technology, Macao, 999078, China

## Abstract

**Background:**

Stable angina pectoris (SAP) is one of the main types of coronary heart disease (CHD). To improve treatment outcomes, more effective biomarkers are needed. Currently, studies on the metabolic characteristics of SAP are lacking. Here, we explored the serum metabolomic profile of SAP and identified potential biomarkers and related pathways to assist the clinical diagnosis and treatment of SAP.

**Method:**

Thirty patients with SAP patients and 30 healthy controls (CON) without stenosis were selected for this study. All patients underwent coronary angiography. The metabolites of the two groups' serum samples were investigated using UHPLC-QE-MS. Changes in serum metabolic profile were evaluated using multivariate statistical analysis and pathway analysis.

**Result:**

OPLS-DA analysis identified significant differences in the serum metabolic profiles between patients with SAP and CON. Twenty-five differential metabolites were identified between patients from SAP and CON groups, including choline, creatine, L-arginine, beta-guanidinopropionic acid, isopalmitic acid, xanthine, LysoPC (18 : 1), and LysoPC (20 : 3). Pathway analysis found that these differential metabolites were involved in energy metabolism, oxidative stress, purine metabolism, and other metabolic pathways.

**Conclusion:**

By comparing the serum metabolic profiles of SAP patients with a control group, we identified 25 potential biomarkers that could improve the clinical diagnosis and treatment of SAP.

## 1. Introduction

Ischemic heart disease is among the most common and most lethal causes of heart failure [1]. According to the Global Cardiovascular Burden Report statistics, 197 million patients were diagnosed with ischemic cardiomyopathy worldwide in 2019, and the burden of ischemic heart disease is increasing annually [2]. Coronary heart disease (CHD) is associated with a severe burden on the global population's health and economy, and its age of onset is gradually getting younger ([3].

At present, coronary angiography is the gold standard for diagnosing CHD, but many patients are reluctant to undergo this examination due to its invasiveness [4]. Therefore, more research on the prevention, early diagnosis, and treatment of CHD are needed. The discovery of new biomarkers has been an important research focus to achieve this.

Technical advances have allowed researchers to use techniques such as genomics, proteomics, and metabolomics to efficiently characterize individuals of a particular disease. Metabolomics is an approach that examines low-molecular weight metabolites (<1,000 Da) of an intact tissue or biofluid in a patient [5, 6] and has been used in patients with CHD [7–9]. The three general metabolomics technologies are nuclear magnetic resonance spectroscopy, gas chromatography-mass spectrometry, and liquid chromatography-mass spectrometry. Their use has brought new opportunities for the study of biomarkers in CHD, such as lysophosphatidylethanolamine, monoglyceride [10], docosapentadilute acid [11], unsaturated fatty acid [12], phenylacetylglutamine [13], and amino acid [14]. However, there are few metabonomic markers that can be used in the clinical diagnosis of CHD. The existing ones have the following disadvantages. First, there were several inconsistencies in the metabonomic methodologies used and pretreatment sample loading used in each study, and the detection ability of metabolites has been shown to vary with different instruments and methods. Second, many predictive biomarkers found in current research are difficult to be clinically validated due to challenges for obtaining endogenous metabolite standards. Thus, despite current advances, more studies with standard methodologies should be performed and validated to assist in the diagnosis and treatment of CHD.

In this study, we used UHPLC-QE-MS technology to detect the serum metabolomics of patients with stable angina pectoris (SAP) to identify potential biomarkers that could guide the diagnosis and treatment of SAP.

## 2. Materials and Methods

### 2.1. Patients and Study Criteria

From March 2021 to September 2021, a total of 60 participants who were treated at the Affiliated Traditional Chinese Medicine Hospital of Southwest Medical University (Sichuan, China) were enrolled. Patients with SAP diagnosed by coronary angiography were arranged into the SAP group, while those with no stenosis confirmed by coronary angiography were selected as the control group (CON). The diagnostic criteria of SAP was performed in accordance with *Nomenclature and Criteria for Diagnosis of Ischemic Heart Disease*, issued by Joint International Society and Federation of Cardiology/World Health Organization in 1979.

The study inclusion criteria were as follows: (1) patients aged from 40 to 80 years; (2) previous coronary angiography showed that at least one coronary artery met the following conditions: 50% ≤ main coronary artery stenosis <75% or 50% ≤ branch coronary artery stenosis <100%; and (3) patients that were to be in the CON group had to have matched basic information in terms of gender, culture, and education with those from the SAP group. The patients were excluded if they had (1) chest pain caused by neurosis, climacteric syndrome, cervical spondylosis, gastric, esophageal reflux, unstable angina pectoris, myocardial infarction, cardiomyopathy, and other diseases; (2) myocardial infarction (at least three months before enrollment) and preinfarction symptoms several months before the study; (3) severe heart failure and malignant arrhythmia affecting hemodynamics; (4) other severe systemic diseases such as AIDS, malignancy, gastrointestinal bleeding, gastric ulcer, and bleeding tendency; (5) liver and kidney dysfunction caused by noncardiac causes; (6) valvular heart disease, congenital heart disease, and active myocarditis without operation; (7) planned pregnancy, were pregnant, or lactating; (8) a history of primary organ (i.e., lung, liver, heart, bone marrow, kidney) transplantation; (9) psychological problems; and (10) participated in other clinical researchers in the recent two months.

All patients and their families gave informed and signed consent for the anonymous use of their data. This study was approved by the ethics committee of the Affiliated Traditional Chinese Medicine Hospital of Southwest Medical University (No. KY20210008-FS01).

### 2.2. Sample Collection

After fasting, 5 mL of venous blood was collected between 7 : 00 and 8: 00 am, placed in 25°C for 30 min, and centrifuged at 3000 rpm for 10 min, and then, 500 *μ*L of the supernatant was transferred to a cryopreservation tube. After liquid nitrogen quick freezing, it was stored in a refrigerator at −80°C until measurement and experimenting purposes.

### 2.3. Sample Preparation

First, 50 *μ*L of the sample was placed into an EP tube, to which 150 *μ*L extract (100% methanol, containing isotope-labeled internal standards mixture) was added, vortexed for 30 s, sonicated for 10 min (ice water bath), and incubated for 1 h at -40°C. Second, the sample was centrifuged at 12,000 rpm for 15 min at 4°C, after which the supernatant was taken to a fresh glass vial for analysis. The quality control (QC) sample was prepared by mixing an equal aliquot of the supernatants from all samples.

### 2.4. Metabolomics Study

The reference of the experiment method is “Optimization and Testing of Mass Spectral Library Search Algorithms for Compound Identification” [15]. UHPLC-QE-MS analyses were performed using the UHPLC system (Vanquish, Thermo Fisher Scientific) coupled to Q Exactive HFX mass spectrometer (Orbitrap MS, Thermo). Chromatographic analysis was performed using an UPLC HSS T3 (2.1 mm ×100 mm, 1.8 *μ*m). The mobile phase consisted of 5 mmol/L of ammonium acetate and 5 mmol/L of acetic acid in water (A) and acetonitrile (B). The analysis was carried with elution gradient using the following steps: 0-0.7 min, 1% B; 0.7-9.5 min, 1%-99% B; 9.5-11.8 min, 99% B; 11.8-12.0 min, 99%-1% B; and 12-14.8 min, 1% B. The column temperature was kept at 35°C. The autosampler temperature was 4°C, and the injection volume was 3 *μ*L.

All spectra data were acquired using the information-dependent acquisition (IDA) mode by control software (Xcalibur, Thermo, ver: 4.0.27). In the IDA mode, the acquisition software continuously evaluated the full scan MS spectrum. The ESI source conditions were set as follows: sheath gas flow rate as 30 Arb, Aux gas flow rate as 10 Arb, capillary temperature 350°C, full MS resolution as 60000, MS/MS resolution as 7500, collision energy as 10/30/60 in NCE mode, and spray voltage as 4.0 kV (positive) or -3.8 kV (negative), respectively.

To monitor the stability of the UHPLC-QE-MS system, all serum samples were randomized. At the beginning of the sample sequence, two blank samples and one QC sample were injected to confirm that the baseline was stable, and then, QC samples were injected once every ten sample injections.

### 2.5. Statistical Analysis and Data Processing

After the raw data was obtained by the Xcalibur software, they were converted to the mzXML format using ProteoWizard and processed with an in-house program developed using R and based on XCMS for peak discrimination, filtering, alignment, integration, and identification. Then, an Excel file of the preprocessed data was imported into the Simca-p (ver: 16.0.2) software for OPLS-DA analysis, an effective multivariate statistical method that emphasizes global law. It focuses on ignoring the intragroup error and eliminating irrelevant random errors, which maximized the differences among groups in the model. Thus, different metabolites could be identified from the massive data obtained. On the chart, each point referred to a sample and the location of the sample depends on the difference between the metabolites it contains. From the OPLS-DA chart, the degree of aggregation and dispersion of the sample could be assessed. A more aggregated degree referred to the presence of more similar metabolite contents and components in the sample. If it was more dispersed, this referred to a greater difference of metabolite contents and components between different samples. Then, Human Metabolome Database (HMDB) and Metlin were used for metabolites identification, and an in-house MS2 database (BiotreeDB) was used for metabolite annotation. The cutoff for annotation was set at 0.3.

Potential biomarkers were screened according to relevant conditions and were analyzed using hierarchical cluster analysis and correlation analysis. Correlation analysis was used to reveal the synergy between the changes of different metabolites. If the changing trend of certain metabolites was the same, it demonstrated a positive correlation. In contrast, if it was negatively correlated, the degree of correlation between the two variables was expressed by correlation coefficient *r*, with an *r* value between -1 and 1. It could be any value in this range. Positive correlation referred to an *r* value between 0 and 1 and a negative correlation for an *r* value between -1 and 0. The closer the absolute value of *R* to 1 referred to a stronger correlation between the two variables, and a closer absolute value of *R* to 0 represented a weaker correlation between two metabolites.

SPSS software (Statistical Product and Service Solutions, IBM, America, ver: 25.0) was used to test the significance level between the CON and SAP groups; *P* < 0.05 was considered significant.

## 3. Results

### 3.1. Participants Characteristic

In all, 60 patients were eligible for this study, comprising of 30 patients in each group. *t*-tests were used to analyze the data and make comparisons between the 2 groups. There was no statistical difference in terms of sex, age, and laboratory data between the SAP and CON groups (*P* > 0.05). Use of SPSS software. Their demographic and clinical characteristics are illustrated in Table 1.

### 3.2. System Stability

The detection stability was judged by the difference in the peak height of the isotope-labeled internal standard mixture response between the QC samples. As shown in Figure 1, the retention time and response strength of the internal standard in QC samples were stable. We also observed that the instrument data acquisition stability was good.

### 3.3. Differences between the Metabolic Profiles of Patients with Stable Angina Pectoris and Control Subjects

A total of 7124 peaks and 1640 metabolites remained after preprocessing (deviation filtering, missing value filtering, missing value imputation, and data normalization) in both positive and negative modes. Then, the data containing the information of peak number, sample name, and normalized peak area were exported to the SIMCA software package (Sartorius Stedim Data Analytics AB, Umea, Sweden, ver: 16.0.2) for multivariate analysis. The principle component analysis (PCA) demonstrated no significant differences between the SAP and CON groups.

To further compare the difference in serum metabolic profile between the SAP and CON groups, we used orthogonal projections to latent structure-discriminant analysis (OPLS-DA) to analyze the data. The results showed that the difference between the two groups was noticeable (Figure 2). (1) In multivariate analysis, significant projection values greater than 1 (VIP > 1) were used as criteria for differential metabolites. (2) Paired *t*-test was used to compare the relative amount (peak area) of identified metabolites between the two groups (*P* < 0.05) in univariate statistical analysis. The candidate metabolites with VIP > 1 and *P* < 0.05 were considered as differential metabolites between the two groups. Based on the above conditions, a total of 89 significant metabolites were identified through the Human Metabolome Database (HMDB) and Metlin and are presented as filtered results using volcano plot (Figure 3). For a condition of MS2 score > 0.8, 26 differential metabolites were identified as potential biomarkers for SAP.  Table 2 summarizes the detailed information of potential biomarkers.

To better understand the metabolic differences and characterize the metabolites changes between the SAP and CON groups, potential biomarker data were analyzed through hierarchical clustering analysis (Figure 4(a)) and correlation analysis (Figure 4(b)). In the clustering heatmap, increasing expression values are coded with blue to red colors. We observed that 3 metabolites were increased and 23 were decreased in the SAP group. Glycoursodeoxycholic acid, FA (20 : 3), and L-arginine were increased, while choline, sphingosine 1-phosphate, beta-guanidinopropionic acid, xanthine, LysoPC (18 : 0), LysoPC (22 : 4), and others were decreased in the SAP group.

### 3.4. Metabolic Pathway Analysis

Metaboanalyst 5.0 was used to investigate the metabolic pathways of the potential biomarkers. The results observed disorder in the glycine, serine and threonine metabolism, arginine and proline metabolism, D-Arginine and D-ornithine metabolism, sphingolipid metabolism, glycerophospholipid metabolism, aminoacyl-tRNA biosynthesis, and purine metabolism in SAP group. A summary of the pathway analysis is shown in Figure 5.

## 4. Discussion

Our study identified 25 potential biomarkers that were associated with oxidative stress, glucose metabolism, fatty acid metabolism, and amino acid metabolism in the serum of SAP patients. Compared with the CON group, a decreasing trend in isopalmitic acid (IPA), which belong to the monomethyl branched-chain fatty acid (BCFAs) [16], in the SAP group was observed. It was reported that IPA could stimulate peroxisome proliferator-activated receptor alpha (PPAR-*α*) [17]. The activation of PPAR can inhibit the expression of some critical genes, such as nuclear factor kappa B, to regulate and promote inflammation in the vasculature and participate in lipid-lowering and atherosclerosis protection to reduce the risk of cardiovascular disease [18–21]. Thus, lower levels of IPA in the serum of the SAP group could relate to higher levels of inflammation in these patients [22].

Glycosyldeoxycholic acid (GUDCA) is considered to have antiapoptotic, antioxidant, and anti-inflammatory properties [23]. It has been found that GUDCA could reduce the production of lactate dehydrogenase, TNF-*α*, and IL-1*β* in the nervous system and reduce the production of cytochrome C peroxidase in neurodegenerative models [24, 25]. Other studies have found that GUDCA could reduce the development of atherosclerosis, which could be related to GUDCA downregulating the expression of scavenger receptor A1 mRNA, reducing the uptake of oxidized low-density lipoprotein, and inhibiting the formation of macrophage foam cells [26, 27]. However, currently, there are no studies linking GUDCA with the pathophysiology and development of CHD and its subtypes, and this could be a future research direction.

Choline is a precursor of acetylcholine that is essential for lipid metabolism. The main sources of choline were shown to be eggs, milk, fresh vegetables, lean fish, meat, and bread, of which animal food sources were the most important contributors to choline intake [28]. In this study, we found that the level of choline was decreased in the SAP group, compared with the CON group. Studies have shown that plasma choline level in patients with a history of acute myocardial infarction (AMI) was significantly lower than that in patients without a history of AMI [29, 30]. Future studies are needed to explore underlying mechanisms for this observation.

The energy required for normal cardiac function is provided by fatty acid and glucose metabolism. Most ATP is produced by fatty acid (FA) oxidation in cardiomyocytes ([31]. FAs are first catalyzed by acyl-CoA synthetase in the presence of ATP, coenzyme A (COA-SH), and Mg2+ to generate lipoyl CoA, which are then transferred to the mitochondrial matrix for *β*- oxidation [32]. This study found that FA was increased in patients with SAP. The increase of substrate indicates that the oxidation of FAs could be restricted, resulting in a decrease in ATP production and a lack of energy supply in the ischemic myocardium.

The AMPK pathway is the main regulatory pathway of glycometabolism and lipid metabolism and is believed to play a key role in regulating cellular energy. Its activation is believed to promote the production of ATP and inhibit the consumption of ATP. AMPK can be negatively regulated by ACC and activate PFK2 to promote catabolism, such as glycolysis and fatty acid oxidation [33], and increase energy supply. *β*-Guanidinopropionic acid (GPA) is an endogenous AMPK agonist. In recent years, it has been found that GPA can competitively inhibit creatine kinase from reducing blood pressure in rats with essential hypertension [34]. GPA was found to be safe and well-tolerated in human experiments [35]. Other studies have shown that GPA could reduce the rate of mitochondrial oxygen consumption and increase autophagy flux in the cells of skeletal muscle to mitigate the effects of metabolic diseases [36]. However, few GPA studies have been performed for cardiovascular disease, and their correlation remained unknown. In this study, for the first time, we found a significant difference in serum GPA between patients with SAP and controls. However, further studies using larger cohorts of patients should be performed to validate these observations.

LPC is a metabolite of PC. A large prospective epidemiological study showed that LysoPC (18 : 1) and LysoPC (18 : 2) were directly related to the occurrence and development of coronary heart disease [37], and the type of PC was associated with its effect on cardiovascular events [38]. Some studies have shown that S1P had a cardioprotective effect and could protect against ischemic myocardium, which may depend on the activation of RhoA and its downstream protein kinase D. At present, drugs for CHD and ischemia-reperfusion targeting S1P receptor are being developed [39–41]. The decrease in sphingosine 1-phosphate in the SAP group could suggest that the cardioprotective effect of sphingosine 1-phosphate was weakened in these patients.

Despite the promising results observed in this study, some limitations should be highlighted. First, the sample size included in this study was relatively small, and studies with larger clinical sample sizes are needed to confirm our observations further [37, 42]. Second, only patients with SAP were included in the disease group, and the metabolic profiles of several other CHD subtypes were not studied or compared. Third, in regard to the metabolomic analyses, we were not able to conduct a comprehensive qualitative and quantitative analysis of all metabolites since we only collected serum samples and did not collect urine and tissue samples. Further, there more unified and rigorous biological sample collection, and processing specification should have been used, and such could have affected the reliability and repeatability of the experimental results, to a certain extent.

## 5. Conclusion

In this study, we identified 25 potential biomarkers for the clinical diagnosis and treatment of stable angina by comparing and assessing the serum metabolic profiles of patients with SAP. Larger scale, multicenter studies using prospective settings are required to validate these observations.

## Figures and Tables

**Figure 1:** Isotope-labeled internal standards ESI+ and ESI- mode EIC plot of all QC samples (a) and UHPLC-QE-MS detection of ESI+ and ESI- mode TIC plot of QC sample (b).

**Figure 2:** OPLS-DA plot: OPLS-DA score plot showing control samples (CON, red dots, *n* = 30) and stable angina pectoris (SAP, blue dots *n* = 30). (a) Positive mode and (b) negative mode (ESI+: R2X 0.299, R2Y 0.703, Q2 0.0776; ESI-: R2X 0.0888, R2Y 0.888, Q2 0.0217).

**Figure 3:** Volcano plot: each dot in the volcano map represents a metabolite containing all the substances measured in this study. (a) The abscissa represents the multiple changes of the group compared to each substance (the logarithm based on 2), and the ordinate represents the *P* value of the Student's *t*-test (the negative logarithm based on 10). (b) The size of dots represents the VIP value of OPLS-DA model (the larger the dot, the larger the VIP value; upregulated metabolites in red, downregulated metabolites in blue, and nonsignificant metabolites in gray).

**Figure 4:** Correlation analysis and clustering heatmap of potential biomarkers in serum. (a) Heatmap of hierarchical clustering analysis of the metabolites determined from serum samples (increasing expression values are coded with blue to red colors. Rows indicate potential biomarkers; columns indicate different groups). (b) Heatmap of correlation analysis of the metabolites determined from serum samples. The rows and columns represent the different metabolites compared in this group. The color blocks at different positions represent the correlation coefficient between the metabolites at corresponding positions. Red represents positive correlation, and blue represents negative correlation; the darker the color, the stronger the correlation. Meanwhile, the significance in correlation was marked with an asterisk.

**Figure 5:** Pathway analysis: (a) Glycine, serine, and threonine metabolism; (b) arginine and proline metabolism; (c) D-Arginine and D-ornithine metabolism; (d) caffeine metabolism; (e) sphingolipid metabolism; (f) glycerophospholipid metabolism; (g) aminoacyl-tRNA biosynthesis; and (h) purine metabolism.

**Table 1:** Demographic and clinical characteristics of the subjects between the two groups.

Characteristics	SAP group (*n* = 30)	CON group (*n* = 30)	*χ* ^2^/*T*	*P* value
Sex				
Male (*N*, %)	17 (56.67%)	16 (53.33%)	0.067	0.795
Female (*N*, %)	13 (43.33%)	14 (46.67%)		
Age ($\overset{¯}{x}\pm s$, years)	62.3 ± 8.04	58.46 ± 8.99	-1.74	0.087
History of smoking	12(40%)	9(30%)	0.659	0.417
Glu ($\overset{¯}{x}\pm s$, mmol/L)	6.21 ± 1.65	5.41 ± 0.95	-2.312	0.024
TC ($\overset{¯}{x}\pm s$, mmol/L)	4.33 ± 1.24	4.57 ± 0.89	0.87	0.388
TG ($\overset{¯}{x}\pm s$, mmol/L)	1.91 ± 1.11	1.44 ± 1.05	-1.66	0.102
HDL-C ($\overset{¯}{x}\pm s$, mmol/L)	1.26 ± 0.37	1.45 ± 0.32	1.996	0.051
LDL-C ($\overset{¯}{x}\pm s$, mmol/L)	2.66 ± 1.09	2.71 ± 0.18	0.202	0.841
ALT ($\overset{¯}{x}\pm s$, U/L)	22.8 ± 10.9	22.33 ± 10.51	-0.168	0.867
AST ($\overset{¯}{x}\pm s$, U/L)	23.9 ± 9.97	24.13 ± 9.54	0.093	0.927
APO-A ($\overset{¯}{x}\pm s$, g/L)	1.51 ± 0.33	1.65 ± 0.27	1.803	0.077
APO-B ($\overset{¯}{x}\pm s$, g/L)	0.93 ± 0.33	0.99 ± 0.43	0.518	0.606
CR ($\overset{¯}{x}\pm s$, *μ*mol/L)	72.86 ± 15.53	70.86 ± 18.76	-0.450	0.655
UA ($\overset{¯}{x}\pm s$, *μ*mol/L)	326.73 ± 70.59	315.80 ± 69.31	-0.605	0.547
UREA ($\overset{¯}{x}\pm s$, mmol/L)	5.95 ± 1.82	5.37 ± 1.48	-1.333	0.188

Data were expressed as mean ± SD. Glu: glucose; TC: total cholesterol; TG: triglyceride; HDL-C: high-density lipoprotein cholesterol; LDL-C: low-density lipoprotein cholesterol; ALT: alanine transaminase; AST:APO-A: apolipoprotein A; APO-B: apolipoprotein A; CR: creatinine; UA: uric acid; UREA, urea.

**Table 2:** Potential biomarkers in stable angina pectoris based on UHPLC-QE-MS analysis in serum.

Mode	Metabolites	HMDB	RT	*m*/*z*	SAP vs. CON				Trend
					VIP	*P* value	FC	MS2 score	SAP/CON
ESI (+)	Phosphoric acid	HMDB0002142	529.91	98.98	3.68	0.00	0.87	1.00	↓
	Choline	HMDB0000097	556.11	104.11	3.20	0.01	0.88	1.00	↓
	Creatine	HMDB0000064	47.43	132.08	1.42	0.03	0.73	0.99	↓
	Phosphorylcholine	HMDB0001565	542.14	184.07	1.51	0.01	0.89	0.99	↓
	11-beta-Hydroxyandrosterone-3-glucuronide	HMDB0010351	520.70	483.25	1.35	0.04	0.86	0.93	↓
	LysoPC(20 : 3)	HMDB0010393	519.98	546.34	2.48	0.01	0.82	0.93	↓
	LysoPC (18 : 0)	HMDB0010384	606.29	524.37	3.78	0.00	0.81	0.92	↓
	Sphingosine 1-phosphate	HMDB0000277	783.51	380.26	1.86	0.03	0.93	0.90	↓
	Glycoursodeoxycholic acid	HMDB0000708	338.83	450.31	2.28	0.00	1.16	0.89	↑
	LysoPC (22 : 4)	HMDB0010401	561.28	572.37	2.61	0.01	0.76	0.88	↓
	LysoPC (16 : 0)	HMDB0010382	540.32	496.34	3.87	0.00	0.84	0.88	↓
	LysoPC (P-18 : 1(9Z))	HMDB0010408	606.34	506.36	3.47	0.00	0.78	0.84	↓
	LysoPC (20 : 2)	HMDB0010392	560.39	548.37	2.63	0.04	0.87	0.84	↓
	Beta-guanidinopropionic acid	HMDB0013222	65.55	132.08	1.51	0.01	0.74	0.83	↓
	LysoPE (0 : 0/18 : 0)	HMDB0011129	595.80	482.32	2.99	0.04	0.86	0.82	↓
ESI (-)	Isopalmitic acid	HMDB0031068	540.76	255.23	2.46	0.01	0.85	1.00	↓
	Pyruvic acid	HMDB0000243	778.32	87.01	1.87	0.01	0.88	1.00	↓
	FA (20 : 3)	HMDB0060039	655.13	305.25	1.18	0.04	1.21	1.00	↑
	16-Methylheptadecanoic acid	HMDB0031066	606.68	283.26	3.14	0.00	0.84	1.00	↓
	Xanthine	HMDB0000292	95.84	151.03	1.54	0.02	0.83	0.94	↓
	Epsilon-(gamma-glutamyl)-lysine	HMDB0003869	452.61	274.14	1.83	0.04	0.63	0.93	↓
	L-Arginine	HMDB0000517	47.21	173.10	1.49	0.03	1.27	0.92	↑
	LysoPA (18 : 2)	HMDB0007856	519.75	433.24	3.22	0.00	0.78	0.87	↓
	LysoPA (16 : 0)	HMDB0007853	540.77	409.24	3.11	0.00	0.84	0.87	↓
	LysoPC (18 : 1)	HMDB0002815	544.41	580.36	2.24	0.01	0.85	0.86	↓
	LysoPC (16 : 0)	HMDB0010382	528.80	554.35	3.30	0.00	0.80	0.86	↓

## Data Availability

The data used to support the findings of this study are available from the corresponding author upon request.
